The article "Clinical Efficacy of Topical Tacrolimus on Conjunctival Hyperemia Caused by Prostaglandin Analogues" was retracted in 2023. Reasons: signs of a paper mill; suspected computer-generated content; unreliable results or conclusions; concerns about the data.

# Clinical Efficacy of Topical Tacrolimus on Conjunctival Hyperemia Caused by Prostaglandin Analogues

**DOI:** 10.1155/2022/3700720

**Published:** 2022-10-14

**Authors:** Jing Yang, Yiyu Shi, Haibo Chen

**Affiliations:** ^1^Hainan Eye Hospital and Key Laboratory of Ophthalmology, Zhongshan Ophthalmic Center, Sun Yat-sen University, Haikou, Hainan 570311, China; ^2^Department of Ophthalmology, Hainan Aier Ehope Eye Hospital, Haikou 570226, China

## Abstract

**Objective:**

To evaluate the clinical efficacy of tacrolimus ophthalmic solution on conjunctival hyperemia caused by prostaglandin analogues.

**Methods:**

A retrospective analysis was performed on 120 patients diagnosed with bilateral primary open-angle glaucoma (POAG). The enrolled patients developed symptoms of conjunctival hyperemia during the administration of travoprost ophthalmic solution. The patients were divided into two groups: 0.004% travoprost solution was administered in the control group. A combination of 0.004% travoprost solution with tacrolimus was administered in the experimental group. Clinopathological parameters including intraocular pressure (IOP), subjective dry eye symptom score (SDES), hyperemia score, and noninvasive tear break-up time (NIBUT) were recorded at week 0, 1, 2, and 4. Two-way ANOVA for repeated measurement was employed for statistical analysis using SPSS 22.0 software.

**Results:**

At week 1, 2, and 4, the IOP and SDES of both the control and experimental groups were significantly lower when compared the values at week 0 (before treatment). No significant differences in the IOP values between the two groups were observed at all time points. At week 2, the SDES and hyperemia score were lower in the experimental group than those in the control group, and the NIBUT was significantly longer in the experimental group. The above parameters showed no significant difference at week 4 between the two groups, although the average SDES and hyperemia score were slightly lower in the experimental group.

**Conclusion:**

Tacrolimus ophthalmic solution can relieve conjunctival hyperemia, improve ocular surface conditions, and reduce discomfort caused by prostaglandin analogues.

## 1. Introduction

Glaucoma is the second most common eye disease which can eventually lead to blindness [1]. The increased intraocular pressure (IOP) is a major risk factor associated with the progression of glaucoma. Since the effectiveness of the optic neuroprotective therapy is uncertain [2], the main therapeutic goal in glaucoma treatment is to lower IOP, reduce retinal ganglion cell loss, and maintain the visual function. There are different strategies to lower IOP [3]. Prostaglandin analogues (PGAs) are the main therapeutic to reduce IOP in glaucoma patients, which shows a good IOP-lowering effect at daily dosing frequency [4, 5]. However, these drugs cause side effects such as conjunctival hyperemia, eyelash elongation, eyelid, and iris pigmentation [6, 7]. Conjunctival hyperemia appears to be a major symptom at the early stage of PGA administration, which impinges on the eye vision and patients' compliance with medication [8, 9]. At present, there are no effective strategies to ameliorate conjunctival hyperemia caused by PGAs.

Tacrolimus (also known as FK506) is a fermentation product isolated from *Streptomyces tsukubaensis* and belongs to macrolide antibiotics [10]. It is a powerful immunosuppressant commonly used in transplantation, which acts by inhibiting the release of interleukin-2 (L-2) and the activation of T lymphocytes [11, 12]. Topical tacrolimus have been reported to show beneficial effects in inflammatory and allergic eye diseases [13, 14]. Since conjunctival hyperemia is usually triggered by microvasculature vasodilation upon inflammatory responses [15, 16], it is plausible that tacrolimus may alleviate the inflammatory conditions in conjunctival hyperemia caused by PGAs.

In this study, a total number of 120 patients diagnosed with POAG and developed the symptoms of conjunctival hyperemia after PGA administration were randomly divided into the control group (0.004% travoprost solution) and the experimental group (a combination of 0.004% travoprost solution with tacrolimus). The ocular parameters including intraocular pressure (IOP), subjective dry eye symptom score (SDES), hyperemia score, and noninvasive tear break-up time (NIBUT) were followed for 4 weeks after treatment. We found that the administration of tacrolimus ophthalmic solution can relieve conjunctival hyperemia and reduce eye discomfort. Our data suggest that topical tacrolimus administration can serve as a potential strategy for alleviating conjunctival hyperemia induced by PGAs.

## 2. Subjects and Methods

### 2.1. Subjects

A total number of 120 patients (65 men and 55 women) who had been diagnosed with bilateral primary open angle glaucoma (POAG) and developed conjunctival hyperemia after 3–5 days' treatment of travoprost ophthalmic solution were enrolled in the study. This was a single-blinded study in which the medical staffs were aware of the treatment while the patients were not informed of the details of the medication. The patients' ages ranged between 28 and 67 years, with an average age at 50.3 ± 8.9 years (mean ± SD). The diagnostic criteria for POAG were based on the Chinese Glaucoma Guidelines (2020) [17]. All those patients had not been treated by any other medications and did not have any medical records of PGA-treated hyperemia before the enrollment in the study. Patients with other immunological disorders, ocular surface diseases, or who had undergone ocular surgery were excluded from the analysis. This study was approved by ethical committee of our hospital and all the enrolled patients signed an informed consent.

### 2.2. Methods

The patients were randomly assigned into the control and experimental groups (*n* = 60 in each group). Fisher's randomization technique was employed for random assignment [18]. All the enrolled patients suffered from conjunctival hyperemia within 5 days after topical application of 0.004% travoprost ophthalmic solution (TRAVATAN *Z* ophthalmic solution 0.004%, Alcon Laboratories Inc., 200 *μ*L/per eye, once a day at 9 : 00 pm). Patients in the control group continued to be treated with travoprost ophthalmic solution only; while patients in the experimental group received a mixture of travoprost solution and tacrolimus, with travoprost ophthalmic solution at final concentration of 0.004%, and Talymus ophthalmic solution at final concentration of 0.1% (Senju Pharmaceutical Co., Ltd). All the solutions were administrated 200 *μ*L/per eye, 4 times a day.

### 2.3. Observation Indexes

Intraocular pressure (IOP) : IOP was measured by a Goldmann tonometer for 3 times at each time point, and the average value was recorded as the IOP.

Subjective dry eye symptoms score (SDES) : SDES was assessed by questionnaire on week 0, 1, 2, and 4. The scoring criteria: Score 0: no dryness, foreign body sensation and burning sensation; Score 1: occasional occurrence of the above symptoms; Score 2: intermittent occurrence of the above symptoms; Score 3: persistent occurrence of the above symptoms. The scores of the patients in each group were summed at each time point and divided by the total number of patients as SDES.

Ocular redness index and noninvasive tear film break-up time (NIBUT) : the ocular redness index and NIBUT were measured by Oculus Keratograph.

### 2.4. Statistical Analysis

SPSS 22.0 was used for statistical analysis, and data were summarized as mean ± standard deviation. Two-way ANOVA for repeated measurement was used for the statistical comparison between the two groups, with Tukey's test as the post hoc test. *P* < 0.05 was considered to be statistically significant.

## 3. Results

After treatment with travoprost ophthalmic solution for 1 week, patients in both the groups showed typical symptoms of conjunctival hyperemia (see Figure 1) and high conjunctival index (see Figure 2). In the experimental groups administrated with tacrolimus ophthalmic solution, the symptoms of conjunctival hyperemia and high conjunctival index were significantly ameliorated after 3 weeks (see Figure 3 and Figure 4).

IOP: compared with week 0 (before travoprost ophthalmic solution and tacrolimus ophthalmic solution treatment), the IOP values at week 1, 2, and 4 were significantly reduced in both the groups (*P* < 0.05). However, there was no significant difference between IPO values of the two groups at all time points (*P* < 0.05) (Table 1).

SDES : compared with week 0, the SDES values at week 1, 2, and 4 were significantly higher in both the groups (*P* < 0.05). At week 0 and week 1, there were no statistical differences in the SDES between the two groups. However, at week 2 the SDES in the experimental group was significantly lower than that of the control group (*P* < 0.05) (Table 1). At week 4, the SDES was also slightly lower in the experimental group, although the difference between the two groups was not significant (*P* > 0.05).

Hyperemia score: compared with week 0, hyperemia scores at week 1 and 2 were significantly higher in both the groups (*P* < 0.05). At week 0, 1, and 4, hyperemia scores remained at a similar level between the two groups. At week 2, the hyperemia score in the experimental group was significantly lower than that of the control group (*P* < 0.05) (Table 1).

NIBUT : compared with week 0, NIBUT values at week 1 and 2 were significantly lower in both the groups (*P* < 0.05). No statistical differences in NIBUT were observed between the two groups at week 0, 1, and 4. At week 2, NIBUT was significantly longer in the experimental group (*P* < 0.05) (Table 1).

1. Indicates *p* < 0.05 when compared to the value at week 0.
2. Indicates *p* < 0.05 when compared to the control group.

## 4. Discussion

Lowering the IOP by medication is an effective treatment for patients with hypertension or primary open-angle glaucoma [3]. Nonadherence to glaucoma eye treatment is a significant barrier limiting the treatment outcome in glaucoma patients. Medication compliance depends on many factors, such as the cost, convenience, and side effects [19,20]. Prostaglandin analogues (PGAs) are a class of unsaturated fatty acids derived from arachidonic acid in the cyclooxygenase pathway. PGAs are able to reduce the IOP by increasing the blood flow in retinal vasculatures and nursing the optic nerve in the retina [21]. In clinical practice, prostaglandins and its analogues are widely used to lower the IOP in glaucoma patients.

The administration of PGAs is accompanied by local side effects, such as conjunctival hyperemia, eyelash elongation and eyelid pigmentation [22]. It has been suggested that conjunctival hyperemia after PGA administration can be triggered by the preservative in the solution [22], since better ocular tolerance was observed when the patients were treated with preservative-free latanoprost. Experimental evidence indicates that latanoprost, which contains the highest concentration of benzalkonium chloride, seems to result in a lower incidence of conjunctival hyperemia [23].

The onset of conjunctival hyperemia involves conjunctival vasodilation, which is mediated by intracellular calcium and endothelium-derived nitric oxide [24]. However, recent evidence also suggests that conjunctival hyperemia can be induced by ocular vasodilation due to infectionor noninfectious agents [15,16]. Tacrolimus functions as a calcineurin inhibitor and is widely as an immunosuppressant in transplantation [14,25]. Since calcineurin is calcium-dependent phosphatase involved in the activation of immune responses [26], we attempted to investigate its potential effect on the conjunctival hyperemia caused by PGAs. Although tacrolimus ophthalmic solution showed no significant effect on the IOP, the administration of tacrolimus improved the ocular surface condition, alleviated subjective dry eye symptom and hyperemia, and prolonged noninvasive tear break-up time after 2 weeks. However, there was no significant difference observed at week 4 between the two groups, although the average SDES and hyperemia score in the experimental group were slightly lower. We reasoned that the patients became adapted to the PGA treatment gradually, and the conjunctival hyperemia improved itself without tacrolimus treatment at week 4. This can also be evidenced by the observation that, at week 4 the hyperemia score and NIBUT became comparable to those of week 0 (before treatment) in both the groups. Overall, these data suggest that the administration of tacrolimus produces a temporary or short-term relieving effect on conjunctival hyperemia caused by PGAs. We also found that some patients developed intolerable hyperemia after the long-term use of PGAs. After tacrolimus medication, the symptoms of hyperemia were significantly improved and PGA therapy could be continued. It is also worth mentioning that we did not find any side effects or additional symptoms associated with tacrolimus administration.

The preservatives in the ophthalmic solution may have a toxic effect on the ocular surface and induce inflammation [27]. Topical administration of tacrolimus has been reported to show beneficial effects in inflammatory and allergic eye diseases [13,14]. Since conjunctival hyperemia can be induced by pathological retinal vasodilation in response to inflammation [15,16], it is speculated that tacrolimus ophthalmic solution may suppress the inflammatory responses triggered by PGA administration or the preservatives in the solution. However, to what extent the immunosuppressant activity of tacrolimus contributes to its beneficial effects on conjunctival hyperemia needs to be clarified in the future studies.

One of the major limitations of our study is the single-blindness, in which the medical staff were aware of the medication in each group. A double-blinded study design would provide more convincing data by excluding subjective judgment. Moreover, a larger cohort of patients from multiple medical centers would provide more valid conclusion of the effect of tacrolimus on conjunctival hyperemia. In addition, the optimal orders of the administration of tacrolimus and PGAs should be clinically practiced to maximize the treatment outcome.

In conclusion, topical administration of tacrolimus ophthalmic solution can significantly relieve conjunctival hyperemia caused by PGAs in POAG patients. It ameliorates the ocular surface conditions, reduces the discomfort and improves the medication compliance in the patients. Our study provides evidence for the beneficial effect of tacrolimus on conjunctival hyperemia. However, in order to maximize the effect of tacrolimus, the optimal clinical practice of tacrolimus administration together with prostaglandin usage remains to be explored in glaucoma treatment.

## Figures and Tables

**Figure 1:** Conjunctival congestion after travoprost treatment for 1 week.

**Figure 2:** High hyperemia index after 1 week of travoprost treatment.

**Figure 3:** Conjunctival congestion was relieved after tacrolimus treatment for 3 weeks.

**Figure 4:** Hyperemia index decreased after tacrolimus treatment for 3 weeks.

**Table 1:** Comparison of the IOP, SDES, hyperemia score, and NIBUT in the two groups at different time points ($\bar{X}$ ± *s*).

Indexes	Week_0	Week_1	Week_2	Week_4
*Experimental group*				
IOP(mmHg)	26.4 ± 4.1	18.7 ± 3.5^**1)**^	16.2 ± 2.9^**1)**^	16.4±3.7^**1)**^
SDES	0.60 ± 0.51	1.88 ± 0.58^**1)**^	1.41 ± 0.39^**1), 2)**^	1.26±0.29^**1)**^
Hyperemia score	1.02 ± 0.51	2.85 ± 0.56^**1)**^	1.43 ± 0.44^**1), 2)**^	1.25 ± 0.21
NIBUT (s)	13.76 ± 2.51	5.34 ± 2.21^**1)**^	9.43 ± 2.44^**1), 2)**^	11.26 ± 3.29
*Control group*				
IOP(mmHg)	25.2 ± 5.3	19.5 ± 2.9^**1)**^	17.7 ± 3.3^**1)**^	16.9 ± 4.2^**1)**^
SDES	0.70 ± 0.48	1.90 ± 0.74^**1)**^	1.85 ± 0.50^**1)**^	1.33 ± 0.31^**1)**^
Hyperemia score	1.09 ± 0.48	2.96 ± 0.74^**1)**^	2.09 ± 0.56^**1)**^	1.33 ± 0.42
NIBUT (s)	12.89 ± 1.96	5.96 ± 1.99^**1)**^	6.41 ± 1.56^**1)**^	10.69 ± 3.42

## Data Availability

All data used in this study are presented in the manuscript.

## Additional Points

Topical tacrolimus administration improves the SDES and hyperemia score in POAG patients. Topical tacrolimus administration does not affect the IOP values in POAG patients. Topical tacrolimus administration reduces discomfort in POAG patients.
